The article "Sports Economic Operation Index Prediction Model Based on Deep Learning and Ensemble Learning" was retracted in 2023. Reasons: unreliable results or conclusions; concerns about the data; concerns about the peer review; concerns about the citations.

# Sports Economic Operation Index Prediction Model Based on Deep Learning and Ensemble Learning

**DOI:** 10.1155/2022/9085349

**Published:** 2022-03-28

**Authors:** Chuangjian Yang, Junmeng Chen

**Affiliations:** ^1^School of Physical Education and Health, East China Jiaotong University, Nanchang 330013, China; ^2^Sangmyung University, Seoul 03016, Republic of Korea

## Abstract

In order to construct a prediction model of sports economic operation indicators, this paper combines deep learning and ensemble learning algorithms to integrate and improve the algorithms and analyzes the principles of the LightGBM ensemble learning model and the hyperparameters of the model. Moreover, this paper obtains appropriate intelligent algorithms according to the data analysis requirements of sports economic operation. The break-even analysis method of sports event operation is to find the critical point of the program's profit and loss by analyzing the relationship between the operating cost and profit of the sports event. In addition, this paper uses deep learning and ensemble learning to comprehensively evaluate sports events, constructs a summary evaluation structure of sports items, and evaluates the model in this paper combined with experimental research. The test results verify the reliability of the model in this paper.

## 1. Introduction

With the development of economy and the continuous growth of social material wealth, people began to pursue leisure consumption, and leisure consumption demand gave birth to the leisure industry. The leisure industry refers to the general term for the production of leisure goods and leisure service industries in the national economy triggered by leisure consumption demand [1]. It widely exists in the three major industries of the national economy, including the primary leisure industry, the secondary leisure industry, and the secondary leisure industry. The tertiary industry, of which the tertiary leisure industry is the main industry of the leisure industry, is mainly composed of tourism, culture, sports, and other leisure industries [2]. The transformation of the economic growth mode, especially the consumption-driven economic growth mode, has promoted the rapid development of the leisure industry. Leisure consumption has gradually become a new growth point for the national economy in many countries and regions, and some have even become the dominant region or country [3]. Leisure industries, especially in some tourist cities, have become local pillar industries, and even the economic growth model has shifted from relying on a single leisure subindustry to relying on the overall development of the entire leisure industry. However, the development of China's leisure industry is relatively late, the development of subindustry is unbalanced, tourism and leisure are developing rapidly, out-of-the-box, and the economic effect of the industry is outstanding. The development of cultural leisure and sports leisure is obviously lagging, and the industrial effect is not obvious. This has caused the development of China's leisure industry. The overall level of development and competitiveness is not high; furthermore, tourism and leisure have experienced extensive development for two to three decades, and its development momentum and development space are obviously hindered, which further restricts the growth of China's leisure industry. It is particularly important to explore how to quickly and continuously promote the comprehensive and rapid development of China's leisure industry and make it a new pillar industry of the national economy.

The article "Sports Economic Operation Index Prediction Model Based on Deep Learning and Ensemble Learning" was retracted in 2023. Reasons: unreliable results or conclusions; concerns about the data; concerns about the peer review; concerns about the citations.

The country's economy has taken off, and people's economic consumption levels have also taken a qualitative leap. More and more people have begun to put forward new requirements on their spiritual level, and they have begun to spend their leisure time by improving their aesthetics. Therefore, various top-notch domestic competitions have increasingly become a spiritual demand of people. In recent years, large-scale sports events have become more and more frequent on the world stage. However, the quality of my country's event services is uneven. As an important basis for running sports events, the organizers urgently need to make a big fuss about the quality of event services, because of the excellent service quality of large-scale sports events. Inferiority directly affects the quality and effect of the event. Good service quality will allow participants to continue to support the sport, and poor service quality will make participants feel disgusted and no longer support the sport.

Based on the previously mentioned analysis, this paper combines deep learning and ensemble learning to construct the sports economic operation index prediction model, evaluate the sports economic operation, and provide a reference for the subsequent development of the sports economy.

## 2. Related Work

Literature [4] believes that the distinguishing characteristics of large-scale festivals and ordinary events are as follows: first, this event must attract a large number of participants and viewers, forming a kind of global attention; second, large-scale festivals are also a kind of market strategy; for the tourism industry, especially, it can make organizers and regions receive extremely high attention in the international market; finally, large-scale festivals can create long-term heritage, which can still play a role after the event is over.

The article "Sports Economic Operation Index Prediction Model Based on Deep Learning and Ensemble Learning" was retracted in 2023. Reasons: unreliable results or conclusions; concerns about the data; concerns about the peer review; concerns about the citations.

Literature [5] conducts a systematic literature review of the industry chain efficiency research from the five perspectives of industry chain competitiveness, efficiency (performance), ecological stability, sustainable development capability, and overall effect. Literature [6] adopts the concepts, methods, and means of performance evaluation to realize the process of performance evaluation of the government.

It has become a common phenomenon that sports events drive the development of the tourism industry. Literature [7] believes that hosting sports events can increase the visibility of a city, bring in a large number of visitors, and promote cultural exchanges between cities. Literature [8] explains the specific role of urban characteristics and how sports events shape the unique characteristics of the city and proposes to use the creation of sports events to shape urban characteristics and communicate the distinctive humanistic spirit through tourism. Sports events play an important role in shaping the image of the city and driving the development of the city. Literature [9] believes that the economic effects of sports events lead to the rapid development of urban economy and tourism. Literature [10] proposes that the shaping of sports landscape is also an important means of displaying the culture of the host city, and it has a positive effect on the transmission of the city's image. Literature [11] mentioned the role of sports events in shaping and transmitting the image and brand of the city. Literature [12] proposes that sports events, as one of the most used cultural activities of the city, have a positive impact on the city's image and puts forward five strategies to convey and shape the image of the city.

Literature [13] takes urban sports as a research perspective and establishes a scientific evaluation system for the current situation of urban sports. Literature [14] established a sports rights evaluation system for college students. Literature [15] analyzes the job role and work process of referees and builds an evaluation index system for referee selection. Literature [16] studies sports tourism, gives an evaluation index system for sports tourism human resources, and develops a corresponding evaluation scale. Literature [17] has conducted research from the perspective of economic benefits. The indicators mainly include facility utilization rate, equipment integrity rate, venue revenue, venue self-sufficiency rate, and profit. Literature [18] assesses the economic benefits of stadiums and uses multifactor comprehensive analysis to construct a grading model of stadiums. The literature [19] mainly studies the two basic attributes of venues: “public welfare” and “business.” Literature [20] constructs an evaluation index system for the normal operation of stadium operation and management after sports events are held.

The article "Sports Economic Operation Index Prediction Model Based on Deep Learning and Ensemble Learning" was retracted in 2023. Reasons: unreliable results or conclusions; concerns about the data; concerns about the peer review; concerns about the citations.

## 3. Deep Learning and Ensemble Learning Prediction Algorithm

Ensemble learning is a machine learning technique commonly used in business and economic analysis. Machine learning algorithms usually cannot directly obtain models with better performance in all aspects, while ensemble learning can upgrade multiple weak individual learners with preferences to a strong learner to obtain higher accuracy. The essential idea is to first generate a set of learners, then use strategies to integrate them, and continuously optimize towards the objective function in the iterative process.

The GBDT algorithm consists of a gradient boosting algorithm (gradient boosting) and a decision tree algorithm (decision tree). It uses a decision tree as the base learner, uses the boosting algorithm to combine multiple weak learners into a strong learner through residual fitting, and uses the gradient information from the previous round to construct a decision tree in the iterative process.

### 3.1. Gradient Lifting Algorithm

The idea of the gradient boosting algorithm is an extension of the boosting method. In the iterative process, the loss function is optimized by adding submodels. If the loss function is extended to a differentiable function, and the boosting method and the gradient descent method are combined to obtain the gradient boosting method, the basic idea is as follows.

The formula of the compound model is shown in formula (1), where *f*_*i*_(*X*) is the submodel.

(1) $$\begin{array}{c} F_{m}\left(X\right)=\sum_{i=0}^{m}f_{i}\left(X\right). \end{array}$$

We assume that the loss function is *L*(*Y*, *F*_*m*_(*X*)), use a greedy way to ensure that the loss function is reduced every time a new submodel *f*_*m*_(*X*) is added, and use gradient descent to perform residual fitting.

(2) $$\begin{array}{c} F_{m}\left(X\right)=F_{m-1}\left(X\right)+f_{m}\left(X\right),\\ L\left(Y,F_{m}\left(X\right)\right)<L\left(Y,F_{m-1}\left(X\right)\right). \end{array}$$

### 3.2. Decision Tree Algorithm

The decision tree algorithm uses a tree structure, the root node contains all the samples, the internal nodes represent the feature attribute test, and the leaf nodes are the results of the classification. The learning process of decision tree includes three steps: feature selection, decision tree generation, and pruning. The key point is the division of optimal attributes in the splitting process.

There are three criteria for feature selection: information gain, information gain ratio, and Gini coefficient. Among them, it is commonly used to perform top-down division according to the information gain criterion, and calculate the information gain of each feature during each division and select the maximum value.

The article "Sports Economic Operation Index Prediction Model Based on Deep Learning and Ensemble Learning" was retracted in 2023. Reasons: unreliable results or conclusions; concerns about the data; concerns about the peer review; concerns about the citations.

The information Ent(D) is defined as formula (3), where *P*_*k*_ represents the proportion of the k-th sample in the sample set D.

(3) $$\begin{array}{c} \text{Ent}\left(D\right)=-\sum_{k=1}^{\left|y\right|}p_{k}\log_{2}p_{k}. \end{array}$$

In the information gain formula, *D*^*v*^ represents the value sample contained in the v-th attribute A in the V branch nodes, and the formula is as follows:

(4) $$\begin{array}{c} \text{Gain}\left(D,A\right)=\text{Ent}\left(D\right)-\sum_{v=1}^{V}\frac{\left|D_{v}\right|}{\left|D\right|}\text{Ent}\left(D^{v}\right). \end{array}$$

The decision tree splitting method in the GBDT algorithm is divided into two, one is the method of leaf-wise growth according to the maximum profit, and the other is the method of direct level-wise growth.

According to the way of leaf growth, the required decision tree can be grown with a smaller computational cost. The advantage of this method is that it has high accuracy and can quickly and effectively complete the growth of the tree, but at the same time, it is easy to overfit and the growth process is sequential and cannot be directly accelerated in parallel.  Figure 1 is the process of decision tree growth by leaves.

The way of layer growth means that each node of each layer must be split. Therefore, this method can directly perform parallel acceleration, but it will generate redundant split nodes, which requires a high computational cost. At the same time, each iteration needs to traverse the complete dataset, so higher running memory is required.  Figure 2 is the growth process of a decision tree split by layer.

LightGBM is mainly based on the framework of decision tree algorithms such as GBDT to optimize the use of histogram algorithm, histogram difference optimization, tree growth based on restricted optimal leaf nodes, unilateral gradient sampling, and reordering of category feature histograms. Compared with other decision tree models, it has improved speed, memory consumption, and accuracy.

In order to reduce the computational cost and obtain better accuracy, the LightGBM model uses a tree growth method that splits according to the optimal leaf node. Algorithms can only be executed sequentially in principle, so three methods of feature parallelism, data parallelism, and voting parallelism are used, and parallel acceleration is performed from the three perspectives of feature, data, and communication.

The article "Sports Economic Operation Index Prediction Model Based on Deep Learning and Ensemble Learning" was retracted in 2023. Reasons: unreliable results or conclusions; concerns about the data; concerns about the peer review; concerns about the citations.

#### 3.2.1. Optimization of Histogram Algorithm

The basic idea is to divide continuous feature values into many #bins, use discrete values as indexes, and then search for the best split point on #bin, reducing the computational cost and storage cost. Moreover, the difference optimization of the histogram can be used to further speed up and get better performance. At the same time, due to the discrete nature, LightGBM can naturally handle category features.

The histogram algorithm only needs to store the discretized value #lbin, does not need the original feature value, and does not need to sort. The #bin value can use smaller data types to store training data, such as the uin8_t type, which can reduce memory consumption to 1/8 of the presorting algorithm. The memory optimization process is shown in Figure 3.

#### 3.2.2. Gradient-Based Unilateral Sampling Algorithm (GOSS)

The idea of GOSS algorithm was first applied to the AdaBoost model. The essential idea is to sort the gradients first, retain all instances with large gradients (errors) for sampling, and only randomly sample all instances with small gradients, so as to reduce the amount of information calculation for feature selection in the iterative process. At the same time, in order to reduce the accuracy of the loss, a certain weight value will be given to the small gradient of the sample.

O is the training data set on the fixed node of the decision tree, the instance is {*x*_1_, *x*_2_, ..., *x*_*n*_}, and the gradient of the loss function is denoted as {*g*_1_, *g*_2_, ..., *g*_*n*_}. Then, the traditional calculation of the variance gain of the split feature *j* of the node at *d* is defined as

(5) $$\begin{array}{c} V_{j|O}\left(d\right)=\frac{1}{n_{O}}\left[\frac{{\left(\sum_{\left\{x_{i}\in O;x_{ij}\leq d\right\}}g_{i}\right)}^{2}}{n_{l|O}^{j}\left(d\right)}+\frac{{\left(\sum_{\left\{x_{i}\in O;x_{ij}>d\right\}}g_{i}\right)}^{2}}{n_{r|O}^{j}\left(d\right)}\right]. \end{array}$$

Among them,

(6) $$\begin{array}{c} \left\{\begin{array}{c} n_{O}=\sum I\left[x_{i}\in O\right]\\ n_{l|O}^{j}\left(d\right)=\sum I\left[x_{i}\in O:x_{ij}\leq d\right]\\ n_{r|O}^{j}\left(d\right)=\sum I\left[x_{i}\in O:x_{ij}>d\right] \end{array}\right). \end{array}$$

When using the idea of the GOSS algorithm, the algorithm first sorts the training examples in descending order according to the absolute value of the gradient and composes the instance subset A by the larger gradient *α* × 100%. After that, the algorithm samples the remaining set with a smaller gradient composed of (1 − *a*)  × 100% instances as a subset B of size *b* × |*A*^*c*^|. Finally, the gain ${\tilde{V}}_{j}\left(d\right)$ calculated according to the subset AUB is

(7) $$\begin{array}{c} {\tilde{V}}_{j}\left(d\right)=\frac{1}{n}\left[\frac{{\left(\sum_{\left\{x_{i}\in A_{r}\right\}}g_{i}+1-a/b\sum_{\left\{x_{i}\in B_{r}\right\}}g_{i}\right)}^{2}}{n_{l}^{j}\left(d\right)}+\frac{{\left(\sum_{\left\{x_{i}\in A_{r}\right\}}g_{i}+1-a/b\sum_{\left\{x_{i}\in B_{r}\right\}}g_{i}\right)}^{2}}{n_{r}^{j}\left(d\right)}\right]. \end{array}$$

The definition of each subitem is as follows:

(8) $$\begin{array}{c} \left\{\begin{array}{c} A_{l}=\left\{x_{i}\in A:x_{ij}\leq d\right\},A_{r}=\left\{x_{i}\in A:x_{ij}>d\right\}\\ B_{l}=\left\{x_{i}\in B:x_{ij}\leq d\right\},B_{r}=\left\{x_{i}\in B:x_{ij}>d\right\} \end{array}\right). \end{array}$$

Using the estimated gain ${\tilde{V}}_{j}\left(d\right)$ on a smaller subset of instances instead of the accurate gain ${\tilde{V}}_{j}\left(d\right)$ on all instances to determine the split point can greatly reduce the computational cost. It is proved that GOSS will not lose much training accuracy, but the efficiency is better than random sampling.

The article "Sports Economic Operation Index Prediction Model Based on Deep Learning and Ensemble Learning" was retracted in 2023. Reasons: unreliable results or conclusions; concerns about the data; concerns about the peer review; concerns about the citations.

#### 3.2.3. Mutually Exclusive Sparse Feature Binding

The optimal feature bundling problem can usually use a greedy algorithm to obtain an approximate solution to select the feature values that need to be combined. For the mutually exclusive feature merging process, since the histogram data is discrete, the original data can be distinguished by the offset to achieve the purpose of merging features.

#### 3.2.4. Comparison of LightGBM and XGBoost Models

Compared with another popular ensemble learning framework XGBoost model, the LightGBM model released later has made the following improvements, as shown in Table 1.

The most important parameter settings of the LightGBM model include the learning rate of the algorithm, the maximum depth limit of the decision tree, the number of leaves of a single decision tree, and the selection ratio of features in the iterative process.

The following are the main parameters for control and optimization of the LightGBM model.

(1) mum_leaves is the main parameter that controls the complexity of the tree model, representing the number of leaves per tree. Usually, it is considered that mum_leaves is less than 2mar_sdeph; otherwise, it is easy to cause overfitting problems. Among them, the corresponding relationship between the number of leaves of a full binary tree and the depth of the tree is
  (9) $$\begin{array}{c} \text{num}\_\text{leaves}=2^{\max\_depth}. \end{array}$$
(2) learning_rate is the learning rate of the algorithm. If it is too small, the optimization efficiency of the model will be too low. If it is set too large, it may reduce the accuracy.
(3) max_depth refers to the maximum depth of the tree model, which can prevent overfitting when the data is small.
(4) max_bin is the maximum number of features stored in bin.
(5) min_data_in_leaf is the minimum amount of data that can be set on the leaf, and the small amount of data can also prevent overfitting.
(6) feature_fraction and bagging_fraction are the ratio of selected features to the total number of features and the ratio of selected data to the total data volume respectively. The values of these two parameters are usually between 0 and 1, which can determine the speed of model training and can also deal with overfitting problems.
(7) mm_iterations represents the number of iterations of boosting.

It can be seen that some parameters overlap in improving the accuracy of the algorithm and dealing with the overfitting problem. Therefore, this paper selects the parameters that are relatively important to the model to optimize.

The article "Sports Economic Operation Index Prediction Model Based on Deep Learning and Ensemble Learning" was retracted in 2023. Reasons: unreliable results or conclusions; concerns about the data; concerns about the peer review; concerns about the citations.

We configure parameters to obtain a better model from the balance of training speed, accuracy, and prevention of overfitting. The following are the hyperparameters that have a greater impact on model prediction:

1. improving training speed: increasing learning_rate and decreasing max_bin
2. improving accuracy: increasing max_bin, increasing mum_leaves, and decreasing learning_rate
3. preventing overfitting: limiting the tree depth max_depth and reducing min_data_in_leaf and using smaller mum_leaves

Tuning machine learning model parameters through optimization algorithms is a common research content. After using the particle swarm algorithm to select the hyperparameters of the support vector machine, the optimized support vector machine is applied to the research of power load forecasting, and the optimization ability of the particle swarm algorithm is proved through experiments. However, the algorithm needs to adjust more parameters. Grid tuning is another common method of tuning machine learning model parameters. Through research, Cheng Chen et al. found that the method is relatively single and the parameter improvement range is limited, making it difficult to search for the best on a global scale. Therefore, a new quantum particle swarm algorithm is proposed to optimize the hyperparameters of the XGBoost model. In the research experiment of forecasting marketing data, compared with the XGBoost forecast based on the grid method tuning, the experiment proved that the new model has obtained higher forecast accuracy.

The Drosophila optimization algorithm is an excellent optimization algorithm suitable for machine learning tuning. Its advantages are simple implementation and fewer configuration parameters. The algorithm simulates the characteristics of the fruit fly colony capturing food in the air through smell and first collects various tastes in the air. The fruit flies in the colony obtain the place with the highest concentration of food taste according to their position information, and then, all the fruit flies fly to the smell point. After that, the algorithm also uses the olfactory characteristics of fruit flies to identify the location of the companions and iterates again, using the olfactory and visual characteristics of fruit flies, to gradually find the point with the largest odor concentration in the current area, and obtain the food location, that is, the global approximate optimal solution.

The article "Sports Economic Operation Index Prediction Model Based on Deep Learning and Ensemble Learning" was retracted in 2023. Reasons: unreliable results or conclusions; concerns about the data; concerns about the peer review; concerns about the citations.

Figure 4 is a schematic diagram of the optimization model of the standard fruit fly optimization algorithm.

The standard fruit fly algorithm is simple to implement, and its operation steps are as follows.

**Step 1 .**

The algorithm first initializes the fruit fly population, that is, initializing the population size Sizepop, setting the maximum number of iterations T, and randomly initializing (X_axis, Y_axis) as the initial position of the fruit fly population [21].

(10) $$\begin{array}{c} \left\{\begin{array}{c} X\_axis\;=\text{random}\times \left(\text{top}-\text{bottom}\right)+\text{bottom}\\ Y\_axis\;=\text{random}x\left(\text{top}-\text{bottom}\right)+\text{bottom} \end{array}\right). \end{array}$$

Among them, random is a random number between [0, 1], and top and bottom are the upper and lower bounds of the search interval.

**Step 2 .**

The algorithm generates a random number within a certain range for each individual fruit fly and uses it as the direction and distance of the individual fruit fly in the random search process. The algorithm assigns values to the initialized fruit fly individuals to obtain the next position of the fruit fly. Among them, random value is the search distance.

(11) $$\begin{array}{c} \left\{\begin{array}{c} X_{i}=X\_axis\;+\text{RandomValue}\\ Y_{i}=Y\_axis\;+\text{ Random}x\text{Value} \end{array}\right). \end{array}$$

**Step 3 .**

The algorithm obtains the taste concentration determination value *S*_*i*_ by calculating the distance Dist between the current position of the fruit fly and the origin of the coordinate.

(12) $$\begin{array}{c} {\text{Dist}}_{i}=\sqrt{X_{i}^{2}+Y_{i}^{2}},\\ S_{i}=\frac{1}{Dist_{i}}. \end{array}$$

**Step 4 .**

The algorithm substitutes the obtained *S*_*i*_ into the taste concentration determination function, which is the corresponding fitness function, and calculates the taste concentration Smelli at the individual position of the fruit pupae.

(13) $$\begin{array}{c} {\text{Smell}}_{i}=\text{Function}\left(S_{i}\right). \end{array}$$

**Step 5 .**

The article "Sports Economic Operation Index Prediction Model Based on Deep Learning and Ensemble Learning" was retracted in 2023. Reasons: unreliable results or conclusions; concerns about the data; concerns about the peer review; concerns about the citations.

The algorithm finds the fruit flies with the best odor concentration (take the maximum value as an example) in the current fruit flies population and sets it as the best taste concentration point.

(14) $$\begin{array}{c} \text{bestSmellIndex}=\text{SelectionMax}\left({\text{Smell}}_{i}\right). \end{array}$$

**Step 6 .**

The algorithm judges whether the best taste concentration value is better than the previous best taste concentration. If it is better, the algorithm records the best taste concentration value and the position information bestSmellIndex and makes all fruit flies fly to this position.

(15) $$\begin{array}{c} \left\{\begin{array}{c} X\_axis\;=X\left(\text{bestSmellIndex}\right)\\ Y\_axis\;=\;Y\left(\text{bestSmellIndex}\right) \end{array}\right). \end{array}$$

**Step 7 .**

The algorithm starts iteratively to find the optimal solution. At the same time, it is judged whether the maximum number of iterations set by the algorithm is reached, and the conditions for satisfying other early termination algorithms are obtained. If the current best taste concentration obtained in the iterative process is better than the previous best taste concentration, Step 6 is executed; otherwise, Step 2 to Step 5 is repeatedly executed until the approximate optimal solution is obtained.

The execution flow of the FOA algorithm is shown in Figure 5.

It can be seen from the algorithm execution flowchart that the time required for each optimization of individual fruit flies in the FOA algorithm is T. At the same time, in the iterative process, each individual fruit fly needs to perform a search until the algorithm reaches the maximum number of iterations, so the time complexity of the standard fruit fly optimization algorithm is O(T' × Sizepop). Therefore, the key to the calculation cost of the control algorithm lies in the setting of the maximum number of iterations T and the size of the fruit fly population size.

Prediction evaluation refers to the evaluation of the accuracy of model prediction results or the measurement of prediction accuracy. In statistics, the magnitude of prediction error is commonly used to measure the quality of the prediction effect. Commonly used regression prediction evaluation methods include mean absolute error, mean square error, root mean square error, mean square log error, mean relative error, mean square log error, median absolute error, and coefficient of determination.

*y*_*i*_ is the actual value of a commodity price series, and ${\hat{y}}_{i}$ is the predicted value.

*(1) Mean Absolute Error (MAE)*. MAE is used to describe the difference between the predicted value and the true value. The smaller the value, the better. The average absolute error of *n* samples is as follows:

(16) $$\begin{array}{c} \text{MAE}=\frac{1}{n}\sum_{i=1}^{n}\left|y_{i}-{\hat{y}}_{i}\right|. \end{array}$$

*(2) Mean Square Error (MSE)*. The mean square error is calculated as the square error between the predicted value and the actual value. The MSE of *n* samples is calculated as follows:

(17) $$\begin{array}{c} \text{MAE}=\frac{1}{n}\sum_{i=1}^{n}{\left|y_{i}-{\hat{y}}_{i}\right|}^{2}. \end{array}$$

*(3) Root Mean Square Error (RMSE)*. For the extremely large or extremely small error values in a set of prediction result data, using the root mean square error can well represent the deviation of the prediction result. The calculation is as follows:

(18) $$\begin{array}{c} \text{RMSE}=\sqrt{\frac{1}{n}\sum_{i=1}^{n}{\left(f_{i}-y_{i}\right)}^{2}}. \end{array}$$

*(4) Mean Square Logarithmic Error (MSLE)*.

(19) $$\begin{array}{c} \text{MSLE}=\frac{1}{n}\sum_{i=o}^{n-1}{\left[\log_{e}\left(1+y_{i}\right)-\;\log_{e}\left(1+{\hat{y}}_{i}\right)\right]}^{2}. \end{array}$$

When the target has the characteristics of exponential growth, this indicator is most suitable to use. MSLE is more sensitive to predictions below the true value.

*(5) Median Absolute Error (MedianAE)*. The median absolute error uses the median of all absolute differences between the target and the forecast to calculate the loss, which can reduce the influence of outliers and is defined as

(20) $$\begin{array}{c} \text{Median}AE=\text{median}\left(\left|y_{1}-{\hat{y}}_{1}\right|,...,\left|y_{n}-{\hat{y}}_{n}\right|\right). \end{array}$$

*(6) Coefficient of Determination (R* ^*2*^ *score)*. The best fit between the prediction model and the real data is judged to be 1, and it can be a negative value. The *R*^2^ score of *n* samples is as follows:

(21) $$\begin{array}{c} R^{2}=1-\frac{\sum_{i=1}^{n}{\left(y_{i}-{\hat{y}}_{i}\right)}^{2}}{\sum_{i=1}^{n}{\left(y_{i}-{\bar{y}}_{i}\right)}^{2}}. \end{array}$$

The article "Sports Economic Operation Index Prediction Model Based on Deep Learning and Ensemble Learning" was retracted in 2023. Reasons: unreliable results or conclusions; concerns about the data; concerns about the peer review; concerns about the citations.

## 4. Sports Economic Operation Index Prediction Model Based on Deep Learning and Ensemble Learning

The break-even method is mainly to evaluate the uncertainty of the operating profit of sports events. The break-even analysis method of sports event operation is to find the critical point of the program's profit and loss by analyzing the relationship between the operating cost and profit of the sports event. The procedure for judging the impact of uncertain factors on the economic effects of the sports event operation plan is used to illustrate the degree of risk in the implementation of the sports event operation plan. This critical point is called the break-even point (BEP), as shown in Figure 6.

BEP is the break-even point of sports event operations, *s* is the income from sports event operations, and Q is the numerical value of sports event operation output. Ql is the numerical value of sports event operation output at the point of win-loss balance, *c* is the total cost of sports event operation, and Cr is the cost of sports event operation.

Based on the development standards of China's sports industry, this paper fully considers the general characteristics of the development of the sports industry to construct a first-level indicator system with the guidance of sports industry development theory. The specific content is shown in Figure 7.

This article uses deep learning and ensemble learning to comprehensively evaluate sports events. In the process of comprehensive evaluation, we often use a combination of qualitative and quantitative methods, or the analytic hierarchy process, for comprehensive evaluation. No matter which method or means is adopted, attention must be paid to the validity and reliability of the evaluation. The reason is that the purpose of comprehensive evaluation is ultimately to give an evaluation of whether the decision is feasible or not and the success or failure of sports events. From the previously mentioned main procedure, we can get the procedure of sports event evaluation as shown in Figure 8.

After constructing the above model, we evaluate the effect of the method in this paper. The data of the algorithm in this paper is processed through deep learning and ensemble learning. Therefore, first, the effect of the algorithm in this paper on the processing of sports economic operation indicators data is tested, and the results shown in Table 2 and Figure 9 are obtained.

From the previously mentioned analysis, it can be seen that the method proposed in this paper has a good effect in the data processing of sports economic operation indicators. After that, the prediction effect of the sports economic operation indicators of the model in this paper is evaluated, and the results shown in Table 3 and Figure 10 are obtained.

Through the previously mentioned research, we can see that the sports economic operation index prediction model based on deep learning and ensemble learning proposed in this paper has good results.

## 5. Conclusion

This article attempts to combine China's national conditions and the characteristics of large-scale sports events to construct an index system, which can diagnose and predict various service quality problems existing in the current events, and put forward constructive opinions. The improvement of the service quality of sports events can realize the faster and better development of the urban sports event industry, form a systematic and scientific sports event service quality evaluation system, and provide guidance for the holding of other large-scale sports series events. This article combines deep learning and ensemble learning to construct a sports economic operation index prediction model, evaluate the sports economic operation, and provide a reference for the subsequent development of the sports economy. Through experimental research, it can be known that the sports economic operation index prediction model based on deep learning and ensemble learning proposed in this paper has good results.

The article "Sports Economic Operation Index Prediction Model Based on Deep Learning and Ensemble Learning" was retracted in 2023. Reasons: unreliable results or conclusions; concerns about the data; concerns about the peer review; concerns about the citations.

## Figures and Tables

**Figure 1:** Decision tree divided by leaf growth.

**Figure 2:** Decision tree split by layer.

**Figure 3:** Schematic diagram of LightGBM histogram algorithm memory optimization.

**Figure 4:** Schematic diagram of standard fruit fly optimization algorithm optimization.

**Figure 5:** The execution flow chart of the standard fruit fly algorithm.

**Figure 6:** Break-even analysis.

**Figure 7:** Schematic diagram of the development index of the sports industry.

**Figure 8:** Evaluation program diagram of large-scale sports events.

**Figure 9:** Statistical diagram of data processing effect.

**Figure 10:** Statistical diagram of predictive evaluation of sports economic operation indicators.

**Table 1:** Comparison of the details of the XGBoost and LightGBM models.

Model details	XGBoost	LightGBM
Tree growth pattern	Growth in layers	Growing by leaves restricted by depth
Split point search method	Feature presorting (default)	Histogram algorithm
Income calculation method during split	Data characteristics	Tbin container characteristics
Memory overhead	Big	Small
Categorical characteristics	One-hot encoding	Histogram data processing

**Table 2:** The processing effect of sports economic operation index data.

Number	Data processing	Number	Data processing
1	96.00	17	92.20
2	92.13	18	96.89
3	91.03	19	91.52
4	91.07	20	93.76
5	88.08	21	88.99
6	89.12	22	96.99
7	95.35	23	96.75
8	89.62	24	96.38
9	95.48	25	92.51
10	92.43	26	92.83
11	88.61	27	89.14
12	95.13	28	90.05
13	90.73	29	90.26
14	90.02	30	93.22
15	94.67	31	96.98
16	96.30	32	95.71

**Table 3:** Predictive effects of sports economic operation index.

Number	Predictive evaluation	Number	Predictive evaluation
1	82.28	17	85.66
2	72.06	18	83.94
3	76.29	19	90.39
4	75.24	20	83.28
5	83.70	21	87.51
6	78.22	22	78.75
7	82.70	23	73.14
8	83.94	24	80.76
9	81.57	25	78.83
10	81.81	26	89.52
11	76.04	27	70.32
12	75.05	28	79.77
13	71.66	29	85.16
14	85.97	30	79.83
15	70.54	31	89.47
16	73.19	32	72.08

## Data Availability

The labeled datasets used to support the findings of this study are available from the corresponding author upon request.
